The article "Specific Targeting of Caspase-9/PP2A Interaction as Potential New Anti-Cancer Therapy" was published in 2013. Journal: PLoS One.

# Specific Targeting of Caspase-9/PP2A Interaction as Potential New Anti-Cancer Therapy

**DOI:** 10.1371/journal.pone.0060816

**Published:** 2013-04-23

**Authors:** Issam Arrouss, Fariba Nemati, Fernando Roncal, Marie Wislez, Karim Dorgham, David Vallerand, Nathalie Rabbe, Narjesse Karboul, Françoise Carlotti, Jeronimo Bravo, Dominique Mazier, Didier Decaudin, Angelita Rebollo

**Affiliations:** 1 Inserm UMRS 945, Hôpital Pitié Salpêtrière, Université Pierre et Marie Curie, Paris, France; 2 Laboratory of Preclinical Investigation, Translational Research Department, Institut Curie, Paris, France; 3 Centro Nacional de Biotecnologia, Campus de Cantoblanco, Universidad Autónoma de Madrid, Madrid, Spain; 4 URF Pierre et Marie Curie, Hôpital Tenon, Paris, France; 5 Department of Molecular Cell Biology, Leiden University Medical Center, Leiden, The Netherlands; 6 Instituto de Biomedicina de Valencia, Consejo Superior de Investigaciones Cientificas, Valencia, Spain; 7 Department of Medical Oncology, Institut Curie, Paris, France; University of South Alabama, United States of America

## Abstract

**Purpose:**

PP2A is a serine/threonine phosphatase critical to physiological processes, including apoptosis. Cell penetrating peptides are molecules that can translocate into cells without causing membrane damage. Our goal was to develop cell-penetrating fusion peptides specifically designed to disrupt the caspase-9/PP2A interaction and evaluate their therapeutic potential *in vitro* and *in vivo*.

**Experimental Design:**

We generated a peptide containing a penetrating sequence associated to the interaction motif between human caspase-9 and PP2A (DPT-C9h), in order to target their association. Using tumour cell lines, primary human cells and primary human breast cancer (BC) xenografts, we investigated the capacity of DPT-C9h to provoke apoptosis in vitro and inhibition of tumour growth (TGI) *in vivo*. DPT-C9h was intraperitonealy administered at doses from 1 to 25 mg/kg/day for 5 weeks. Relative Tumour Volume (RTV) was calculated.

**Results:**

We demonstrated that DPT-C9h specifically target caspase-9/PP2A interaction *in vitro* and *in vivo* and induced caspase-9-dependent apoptosis in cancer cell lines. DPT-C9h also induced significant TGI in BC xenografts models. The mouse-specific peptide DPT-C9 also induced TGI in lung (K-Ras model) and breast cancer (PyMT) models. DPT-C9h has a specific effect on transformed B cells isolated from chronic lymphocytic leukemia patients without any effect on primary healthy cells. Finally, neither toxicity nor immunogenic responses were observed.

**Conclusion:**

Using the cell-penetrating peptides blocking caspase-9/PP2A interactions, we have demonstrated that DPT-C9h had a strong therapeutic effect *in vitro* and *in vivo* in mouse models of tumour progression.

## Introduction

Apoptosis is a genetically programmed cell death and its deregulation is associated, among other pathologies, with cancers. Several phosphatases have recently become attractive targets for the treatment of a variety of diseases, including cancers [1], [2], [3], [4]. However, the only clinical drugs targeting a phosphatase are the immunosuppresssive cyclosporin A and FK506, which inhibit Serine/Threonine phosphatase 2B (calcineurin) and NFAT activation [5], [6], [7], [8], [9]. But long-term usage of these drugs can lead to undesirable side effects [10].

The Ser/Thr phosphatases PP1 and PP2A have been implicated both in the induction of cell death through 1) dephosphorylation of Bad [11] and caspase-9 [12] 2) stimulation of cytochrome *c* release [13], and 3) dephosphorylation of the retinoblastoma protein [14], [15]. However, these phosphatases mostly control the phosphorylation level of Bcl-2 and caspase-9, which determines their functional properties [16], [17], [18]. Conversely, the inhibition of PP1[19], PP2A [20], or PP2C [21] triggers cell death, indicating also a potential anti-apoptotic function of these phosphatases, and pointing to a complex interplay of phosphatase actions. We have previously shown an interaction between caspase-9 and PP1α. In this complex, activated PP1α induces caspase-9 dephosphorylation, and as a consequence, its activation leading to apoptosis [12]. We have detected in this complex, in addition to PP1αactivity, another okadaic acid-sensitive enzymatic activity compatible with a PP2A activity, suggesting a possible interaction between caspase-9 and PP2A that may be involved in cell death regulation.

Cell penetrating peptides (CPP) are molecules which can translocate into cells without causing membrane damage, leading to their proposed use as vectors for delivering therapeutic cargo [22]. These peptides can cross the membrane and reach the cytoplasm and/or the nucleus [23]. Using CPP, we have also previously reported experimental evidence as proof of principle for the drug phosphatase technology (DPT), [24], [25].

On these bases, we decided to analyze whether modulation of the PP2A and caspase-9 interaction might have an impact on the induction of tumour cell deathing without effecting healthy cells, and demonstrated DPT-C9h and DPT-C9 corresponding to the binding sites between human and mouse caspase-9 and PP2A respectively, have a specific anti-tumour effect.

## Materials and Methods

### Cells and culture

Human Daudi, Jurkat, and HeLa cell lines were cultured in RPMI supplemented with 10% of FCS. LKR10 and LKR13 have been previously described [26] and were cultured in RPMI supplemented with 10%FCS**.** Human breast cancer (BC), uveal melanoma (UM), non small-cell lung cancer, and small-cell lung cancer cell lines have been isolated from primary human cancer xenografts [27], [28], [29]. The three UM cell lines have been directly obtained from patients’. BC cell lines were cultured in DMEM or RPMI medium supplemented with 10% to 20% of FCS, except for HBCx-15, which was supplemented with 10% of horse serum. UM and lung cancer cell lines were cultured in RPMI supplemented with 10% or 20% of FCS, respectively. The BC and UM cell lines were directly isolated from the corresponding tumor. The Daudi, HeLa and Jurkat cell lines were obtained from the collection of the Department.

### Immunoprecipitation and western blot

The immunoprecipitation and western blot were done as previously described [12]. The anti caspase-9, and anti-PP2A antibodies were purchased from Santa Cruz, Cell Signalling, Sigma or Abcam. The anti-Tim 23 and anti Cyt c were obtained from Transduction Laboratories.

### Peptide synthesis and sequence

Peptides were synthesized as previously described [30].

### Detection of apoptosis by Annexin staining

Apoptosis was detected by Annexin V-FITC staining according to the manufacture’s protocol (BD Bioscience).

### Caspase-9 activity

Caspase-9 activity was detected using the Caspase-Glo 9 kit (Promega) and following the manufacture’s protocol.

### Serum enzyme-linked immunosorbent assay (serum ELISA)

ELISA test was done as previously described [31], [32].

### Miochondrial membrane potential assay

For detection of changes in the mitochondrial membrane potential, we used the Cell Meter JC-10 assay kit following the manufactures’s recommendations.

### Cell cycle analysis

A total of 1×10^6^ cells were fixed in ethanol 70% for 1 h at 4°C. Cells were centrifuged and washed with staining buffer (DPBS/2% FCS). After washing, cells were treated with 50 µl of RNAse (1 mg/ml stock) and incubated for 30 min at 37°C. Cells were stained with 5 µg of propodim iodide for 30 min at room temperature. Cellular DNA content was analyzed by FACS.

### Isolation of Mitochondria fraction

A total of 40×10^6^ cells were washed with chilled PBS. Cell pellet was resuspended in 5 volumes of ice-cold buffer A (20 mM Hepes-KOH, pH 7.5, 10 mM KCl, 1.5 mM MgCl_2_, 1 mM EDTA, 1 mM EGTA, 1 mM DTT, 0.1 mM PMSF, 250 mM sucrose) supplemented with protease inhibitors. Cells were disrupted in a Dounce homogenizer, the nuclei were centrifuged (1000xg, 10 min, 4°C), and the supernatant further centrifuged (10,000xg, 10 min, 4°C), mitochondrial pellet was resuspended in buffer A and stored at –80°C.

### Isolation of cell populations

Fresh blood from healthy donors was collected by the Etablissement Francais du Sang. Chronic lymphocytic leukemia (CLL) samples were obtained from the Hematology Service of the Pitié Salpêtrière hospital. Peripheral blood mononuclear cells (PBMC) isolated from patients or healthy donors were maintained in RPMI 1640 supplemented with 10% FCS, 1% non-essential amino acids, 1% Hepes, 1% sodium pyruvate and 1% glutamine. B cells were isolated using Dynal negative isolation kit (Invitrogene). The purity of the isolated cells reached up to 98%. Human lymphocytes isolated were stained with anti-hCD19-AP and early apoptosis events were determined using Annexin-V-FITC.

### *In vivo* models of primary human tumour xenografts

The primary human breast cancer (BC) xenografts were obtained as previously described [27], [28] Mouse breast cancer tumours were obtained using the transgenic *Polyoma Middle-T* Mouse PyMT model [33]. Spontaneously growing mammary tumours occurring in transgenic mice were xenografted into *nude* immunodeficient mice to allow pharmacological assessments, and maintained from *nude* mouse to *nude* mouse serially passages.

### Mouse model of primary pulmonary adenocarcinoma mutated for *K-ras*

The K-ras^LA1^ mice were provided by the NCI Mouse Models of Human Cancers Consortium (MMHCC) (NCI Mouse Repository/NIH, Rockville, MD). They carry a latent *K-ras* allele with two copies of exon 1: one was the wild-type and the other the G12D mutant (Tyler Jacks). The latent allele is stochastically activated in cells through homologous recombination, which results in deletion of the wild-type copy of exon 1 and the expression of an oncogenic form of the *K-ras* gene. Multifocal lung adenocarcinomas develop spontaneously in 100% of these mice.

### Therapeutic assays

For therapeutic experimental assays in subcutaneous transplanted xenografts (primary human tumours and PyMT tumours), 5- to 8-week old Swiss nu/nu female mice received a subcutaneous graft of tumour fragments with a volume of approximately 15 mm^3^ as previously described [29].

For therapeutic experimental assays in K-ras^LA1^ mice, 16-week old mice were randomized between control (n = 17) or treatment group (n = 16) for 4 weeks. Mice were weighed once a week. At the end of treatment, autopsy was performed for placebo or treatment groups and lung tumours were counted. Results are expressed as tumour number/mouse, mean ± SEM.

Tumour volume was calculated by measuring two perpendicular diameters with calipers. Each tumor volume (v) was calculated according to the following formulae: V = axb^2^/2, where a and b are the largest and the smallest perpendicular tumour diameters. Relative tumour volume (RTV) was calculated from the following formula: RTV = (Vx/V1), where Vx is the tumour volume on day X and V1 is the tumour volume at initiation of the therapy (day 1).Growth curves were obtained by plotting the mean volume of RTV on Y axis against time (X axis, expressed as days after starting of treatment), Antitumor activity was evaluated according to tumour growth-inhibition (TGI), calculated according to the following formulae: percent GI = 100-(RTVt/RTVc)×100, where RTVt is the medium RTV of treated mice and RTVc is the median RTV of controls, both at a given time point when the anti-tumour effect was optimal.

DPT-C9h and DPT-C9 peptides diluted in water/glucose (1 to 25 mg/kg) were given by intraperitoneally route 5 to 7 days per week, according to the models and the therapeutic schedules.

### Bioluminescence assays

HBCx-12A cell line was established from the HBCx-12A xenograft and maintained in RPMI, supplemented with 20% fetal calf serum and penicillin/streptomycin. Cells were transduced with the lentiviral supernatant containing luciferase [19] and Ds-Red and a total of 1.9×10^6^ cells expressing Ds-RED-Luc were implanted subcutaneously into *nude* mice. Growth tumour was measuring by caliper and by optical imaging.

Bioluminescence imaging was performed with the IVIS imaging system (IVIS100, Caliper Life Sciences, USA). Anesthetized mice were injected i.p with luciferin at 150 mg/kg. Imaging acquisition time was from 1 s to 1 min, depending on the bioluminescence signal. Analysis was performed using software Living Image V. 2.50 (Caliper Life Sciences).

### Statistical tests

For *in vivo* experiments’ analyses, statistical significance of differences observed between individual RTVs corresponding to the group of treated mice and the control group, in which 9–10 mice per group have been included, were calculated by a paired Student’s t test [29]. For K-ras^L1^ mice model, we use the Mann Whithney test.

### Peptides sequence

DPT-Sh1: VKKKKIKREIKI

C9: YIETLDGILEQWARSEDL

C9h: YVETLDDIFEQWAHSEDL

DPT-C9h: VKKKKIKREIKI YVETLDDIFEQWAHSEDL

DPC-C9: VKKKKIKREIKI YIETLDGILEQWARSEDL

DPT-C9h Mut: VKKKKIKREIKI YVETLDDIFEQAAHSEDL

All the peptides were solubilised on sterile water.

The experimental protocol and animal housing were in accordance with institutional guidelines as proposed by the French Ethics Committee (Agreement B75-05-18, France). No consent was needed for this study. All surgery was performed under total zylazine/ketamine anesthesia and all efforts were made to minimize suffering.

All patients had previously given their informed consent for experimental research on residual tumour tissue available after histophatologic and cytogenetic analyses. The CLL samples are tumoral residues and the patients given their informed consent. This research was not conducted outside of our country. The ethic committees approve this procedure.

The funders had no role in study design, data collection and analysis, decision to publish or preparation of the manuscript.

## Results

### DPT-C9h peptide blocks the caspase-9/PP2Ac interaction in breast cancer cell lines

We have previously determined the binding site of human and mouse caspase-9 to PP2A (Patent PCT-EP2010/054134, web site: espacenet.com or worlwide.espacenet.com, for peptide sequence, see Materials and Methods) and associated this interaction motif to a cell permeable shuttle [24], [25]. In order to target the caspase-9/PP2Ac interaction, we decided to use the patented peptide containing the previously published penetrating sequence associated to the site of interaction of mouse (DPT-C9) or human (DPT-C9h) caspase-9. As controls, we generated the shuttle DPT-sh1 alone, the peptides C9 and C9h, which did not contain the shuttle and the peptide DPT-C9h mut, with a mutation in the caspase-9/PP2A binding sequence and that does not bind PP2A (data not shown).

We were first interested in confirming that the specific target of DPT-C9h peptide was the complex caspase-9/PP2A. To that end, we analyzed whether the human peptide DPT-C9h wasable to target the *in vivo* and *in vitro* caspase-9/PP2A interaction. For *in vivo* competition, lysates from control untreated or DPT-C9h-treated HBCx-12A cells were immunoprecipitated with anti-caspase-9 antibody and the presence of the caspase-9/PP2A complex was analyzed by western blot. Figure 1A shows that the amount of complex detected in DPT-C9h-treated cells was strongly reduced compared to non-treated control cells. For the *in vitro* competition assay, lysates from HBCx-8 cells were immunoprecipitated with an anti-caspase-9 antibody and the interaction with PP2A competed with the DPT-C9h peptide (Fig 1A). PP2Ac was detected in control caspase-9 immunoprecipitates, while it was almost undetectable after competition with 1.5 mM of DPT-C9h peptide. In both, (*in vitro* and *in vivo* competitions), caspase-9/PP2A complex was not altered by the shuttle DPT-Sh1 (Figure 1B). This strongly suggests that the DPT-C9h peptide specifically targets the interaction between human caspase-9 and PP2Ac.

**Figure 1:** DPT-C9h competes in *in vitro* and *in vivo* caspase-9/PP2Ac interaction. A) *In vivo* competition of caspase-9/PP2Ainteraction. The HBCx-12A breast cancer cell line was cultured for 24 h in the presence or the absence (control) of DPT-C9h (100 µM); cells were lysed and cytoplasmic extracts immunoprecipitated with anti-caspase-9 antibody and immunoblotted with anti-PP2Ac and anti-caspase-9 antibodies. *In vitro* competition of the caspase-9/PP2A interaction. Cytoplasmic lysates from HBCx-12A cells were immunoprecipitated with anti-caspase-9 antibody; the caspase-9/PP2Ac interaction was competed *in vitro* with 1.5 mM of DPT-C9h peptide for 30 min at room temperature; immunoprecipitates were washed and immunoblotted with anti-PP2Ac and anti-caspase-9, the latter as internal control of protein loading. B) The HBCx-12A cell line was cultured in the presence or the absence (control) of the shuttle DPT-Sh1 (100 µM) for 24 h and the *in vitro* and *in vivo* competition of caspase-9/PP2A interaction was analyzed as above.

### The penetrating peptides DPT-C9 and DPT-C9h induce species-specific apoptosis

We analyzed the ability of the two penetrating peptides DPT-C9h and DPT-C9, as well as the negative control peptides C9, C9h and DPT-Sh1 to induce apoptosis. As shown in Figure 2A, DPT-C9h induced apoptosis, as detected by Annexin-V staining in human Daudi, Jurkat, and HeLa cell lines upon 20 h of treatment, whereas the C9 and C9h peptides without shuttle and the shuttle alone, did not induce apoptosis in human cell lines. Similarly, the DPT-C9h peptide did not have any apoptotic effect on the mouse lung cancer cell lines LKR10 and LKR13, while the peptide DPT-C9, specific for mouse caspase-9, induced apoptosis in both cell lines upon 24 h of treatment (Fig 2B). Moreover, we did not observe any apoptotic effect upon treatment of cell lines with the shuttle (Fig 2B). The basal level of apoptosis in non-treated control cells is also shown. These results strongly support species’ specificity for both DPT-C9 and DPT-C9h peptides.

**Figure 2:** DPT-C9h induces apoptosis in human cell lines. **A**) Daudi, Jurkat, and HeLa cell lines were cultured in the presence of DPT-C9h, DPT-Sh1, C9h, or C9 peptides for 20 h at 100 µM and apoptosis was estimated by Annexin-V staining. **B**) Mouse lung cancer cell lines LKR10 and LKR13 were cultured in the presence of DPT-C9h, DPT-C9, or DPT-Sh1 at 100 µM. After 24 h of incubation, apoptosis was estimated by Annexin staining. The basal level of apoptosis of control non-treated cells is shown. P values are also shown (*<0.05; **<0.001; ***<0.0001). **C**) Breast, uveal melanoma and lung cancer cell lines isolated from primary human xenografs were cultured in the presence or absence of DPT-C9h peptide (100 µM) for 24h and apoptosis was estimated by Annexin V-FITC. Basal level of apoptosis without peptide addition is shown (grey colour) p values are shown. **D**). Breast cancer cell lines derived from the primary human xenografts, were incubated with C9h in culture medium at 150 µM and apoptosis induction was estimated at different times. **E**) Breast cancer cell lines isolated from primary human xenografts BCx-3 and Bcx-12 were cultured in the presence or absence (control) of the peptide DPT-C9h for 24 h and apoptosis was estimated.

Using the human breast, uveal melanoma, non-small cell lung and small-cell lung cancer cell lines obtained from primary human xenograft models, we tested the apoptotic effect of both DPT-C9h and C9h peptides. Apoptosis was also analyzed in commercial breast cancer cell lines. In all cell lines analyzed, DPT-C9h induced apoptosis, ranging from 20 to 75% upon 24 h of culture (Fig 2C) while no effect was observed after C9h treatment of breast cancer cell lines (Fig 2D). The apoptosis of the control non-treated cells ranged from 3 to 8%. Supplementary addition of DPT-C9h peptide 27h after the initial treatment strongly increased the level of apoptosis (data not shown). Figure 2E shows two representative apoptosis histogramme plots of two cell lines isolated from the human breast cancer xenograft HBCx-3 and HBCx-12A models treated 24 h with or without (control) DPT-C9h peptide. Taken together, these results show a strong *in vitro* anti-tumoral effect of the DPT-C9h peptide in various human cell lines.

### Inhibition of caspase activity blocks apoptotic effect of DPT-C9h

Given that initiator caspase-9 is an important mediator of apoptosis, we analyzed the ability of DPT-C9h to activate caspase-9 in the human breast cancer cell line HBCx5. Cells were incubated with the peptide and caspase-9 activity was estimated at different times. We have observed an increase of caspase-9 activity in DPT-C9h treated cell line (Fig 3A). Similar results were obtained using cell lines of uveal melanoma and non small cell lung cancer (data not shown). Moreover, using the caspase inhibitor Z-VAD, we observed a decrease in caspase-9 activity.

**Figure 3:** Effect of DPT-C9h on caspase-9 activation, mitochondrial membrane depolarization, cytochrome *c* release and cell cycle. A) HBCx-3 cells were cultured for 3 or 6 h with medium (control), 100 µM of DPT-C9h or 10 µM of the caspase inhibitor Z-VAD (pre incubation of 1h) and 100 µM of DPT-C9h. Caspase-9 activity was estimated using a luminogenic substrate. Results are represented relative to control non-treated cells as arbitrary units. P values are shown. B) HBCx-3 cells were cultured for 24 h with medium (control), DPT-Sh1 (100 µM), DPT-C9h (100 µM) or Z-VAD (10 µM, pre incubation of 1h) and DPT-C9h (100 µM). Apoptosis was estimated by Annexin-V-FITC binding. C) HBCx-3 cells were treated for different periods of time with DPT-C9h (100 µM) and then incubated for 30 min at 37°C protected from the light with the fluorescent probe JC-10. Green and red fluorescence were measured. Data are represented relative to the control non-treated cells. P values are shown. D) HBCx-12A and HBCx-3 cell lines were treated for 24 h with 100 µM of DPT-C9 h. Mitochondrial fraction was separated from whole cell lysates and immunoblotted for cytochrome *c*. The WB was also hybridized with the mitochondrial marker Tim23 as internal control of protein loading. E) HBCx-3 cells were non-treated (control) or treated with 10 or 25 µM of DPT-C9h for 24 or 48 h and the cell cycle was analyzed by FACS.

To determine whether activated caspase-9 is involved in the apoptotic action of DPT-C9h, we analyzed the effect of the caspases inhibitor Z-VAD on cell apoptosis detected by annexin-V-FITC binding. As shown in Fig 3B, the caspase inhibitor markedly reduces apoptosis induced by the peptide. Treatment of the cells with the shuttle or the inhibitor alone does not induce apoptosis (Fig 3B).

### DPT-C9h induces mitochondrial membrane depolarization and cytochrome *c* release without affecting cell cycle

In order to characterize DPT-C9h-induced apoptosis, we investigated the involvement of the mitochondria. In a fluorescence-based assay, the exposure of HBCx-5 cells to peptide induced a marked decrease of the mitochondrial membrane potential (Fig 3C). To confirm the role of mitochondria in DPT-C9h-induced apoptosis, we analyzed whether DPT-C9h treatment induced cytochrome *c* release. Using mitochondrial proteins from control non-treated or peptide-treated cells, we observed the release of cytochrome *c* from the mitochondria in DPT-C9h treated cells while in non-treated control cells, cytochrome *c* is retained in the mitochondrial fraction (Fig 3D). The ratio of cytochrome *c*/Tim 23 is used as internal control for normalization and quantification of the amount of liberated Cyt *c.* These results confirm the mitochondrial implication in DPT-C9h-induced apoptosis.

Finally, we analyzed whether DPT-C9h peptide could interfere in the cell cycle sequence. Cells were non-treated (control) or treated with different doses of peptide for different periods of times and cell cycle distribution was analyzed (Fig 3E). Using *in vitro* sub-apoptotic dose of peptide, we showed that DPT-C9h did not induce accumulation of tumour cells in any phase of the cell cycle, whatever concentration used and time analyzed (Fig 3E).

### DPT-C9h has effect on tumoural cells, but not on healthy cells

Chronic lymphocytic leukaemia (CLL) is characterized by accumulation of monoclonal B cells CD5+ in hematopoietic organs, which reflects a defect in apoptosis. In order to evaluate the apoptotic effect of DPT-C9h peptide in primary healthy and tumour cells of similar origin, we used peripheral blood mononuclear cells (PBMC) from healthy donors and chronic lymphocytic leukaemia patients (CLL). PBMC from healthy donors or CLL patients were treated for 3h with DPT-C9h peptide, washed, resuspended in complete medium without peptide for 6h and then analyzed for apoptosis. Fig 4A shows that DPT-C9h has an apoptotic effect on B cells from CLL patients but not on B cells from healthy donors relative to control non treated cells. DPT-C9h has no effect on T, NK and monocytes from healthy donors or CLL patients. The shuttle DPT-Sh1 or C9h peptides alone had no effect (data not shown). Finally, a similar pro-apoptotic effect of DPT-C9h peptide was observed when B cells were isolated from bone marrow of CLL patients (Fig 4B). This result strongly suggests that only tumour B cells are affected by DPT-C9h treatment without any effect on cells from healthy donors, underscoring the specific tumoural effect of DPT-C9h.

**Figure 4:** Apoptotic effect of DPT-C9h peptide on primary and tumour cells. **A**) Peripheral blood mononuclear cells (PBMC) from healthy donors or CLL patients were cultured in the presence of DPT-C9h (150 µM) for 3 h, then washed, transferred to complete medium and apoptosis was estimated 6h later. Selection of B cells was done by anti-CD19 antibody before Annexin V-FITC staining. Non-treated cells were used as control. **B**) Cells isolated from bone marrow of CLL patients and healthy donors were treated as in A and analyzed for apoptosis. P values are shown.

### Lack of immunogenic activity and *in vivo* toxicity of DPT-C9h and DPT-C9 peptides

Given that our final interest is to prove an anti-tumour effect of DPT-C9h on human cancers, we decided to analyze the *in vivo* immunogenic activity of the peptide. *Nude* immunodeficient T-cell mice were treated five days per week during 6 weeks by intraperitoneal injections of DPT-C9h. Sera were collected at different times and the production of antibodies directed against DPT-C9h or DPT-Sh1 was analyzed. Using ELISA test, we did not detect any in the antibodies against DPT-C9h or DPT-Sh1 throughout the kinetic analyzed at two different doses of peptide (Fig 5A). Similarly, the antibody response was also analyzed using immunocompetent mice, again showing lack of antibody production neither against DPT-C9h nor DPT-Sh1 peptides (Fig 5B). This result strongly suggests that the DPT-C9h peptide is immunogenic even after prolonged *in vivo* administration in immunocompetent or immunodefficient mouse models.

**Figure 5:** *In vivo* antibody responses and toxicity induced by DPT-C9h. **A** ****) Serum antibodies taken from nude mice treated for different periods of time were detected by ELISA at two different concentrations of DPT-C9h peptide (10 and 50 µM). **B**) Serum antibodies from wild type mice treated for different periods for time were tested by ELISA against DPT-C9h and DPT-Sh1 (50 µM). **C**) DPT-C9h was intraperitoneally administered in mice bearing tumors HBCx-12A at 1, 5, or 25 mg/kg once daily for 5 weeks; the median weight of mice for each experimental group is represented at different times. A total of 10 mice were included per group. Similarly, DPT-C9h was intraperitoneally administered in mice bearing tumours HBCx-8 at 10 mg/kg twice daily for 4 weeks. DPT-C9 was IP administrated at mice model PyMT model at dose of 5 mg/kg. The median weight of mice for each experimental group is represented at different times. Ten mice were included per group.

Before *in vivo* therapeutic assessment, the toxicity of DPT-C9h was evaluated in mice bearing HBCx-8 and HBCx-12A tumours after various schedules of administration, i.e. intraperitoneal injections at 1, 5, or 25, mg/kg once daily, or 10 mg/kg twice daily, for 4 to 5 weeks. Whatever the dose, we did not observed any side effects in all treated mice, as well as a complete weight stability of the treated mice (Fig 5C). In addition, no death was observed throughout the experiment. Finally, to confirm the absence of toxicity of the mouse specific peptide, we evaluated tolerability of the DPT-C9 peptide administered at 5 mg/kg once daily in the transgenic *Polyoma Middle-T* Mice PyMT (Fig 5C). In all experiments, no side effects, including weight loss were observed.

### DPT-C9h and DPT-C9 induce *in vivo* inhibition tumour growth in lung and breast cancer models

To first confirm the *in vivo* induction of species-specific apoptosis, we evaluated the efficacy of the DPT-C9 peptide in the K-ras^LA1^ adenocarcinoma mouse model and in transgenic *Polyoma Middle-T* Mice (PyMT). Administered intraperitoneally at a dose of 5 mg/kg for 5 days/7 for 4 weeks, DTC-C9 induced a significant decrease in lung tumour burden as the number of tumours per mouse was 24.6±2.8 (mean±SEM) in the placebo group compared to 15.4±1.9 in the treated group (p = 0.01) (Fig 6A). Figure 6B shows the histological analysis of lung tissue of control and DPT-C9h-treated representative mice. Moreover, *Nude* mice bearing xenografted mouse PyMT breast tumours were treated intraperitoneally with the mouse-specific DPT-C9 peptide at a daily dose of 5 mg/kg. Despite a very fast spontaneously tumor growth, DPT-C9 induced a significant TGI of 46% (p<0.03) (Fig 6C). The relative tumour volume (RTV) was calculated as described in detail in Materials and Methods.

**Figure 6:** *In vivo* therapeutic efficacy of DPT-C9 and DPT-C9h. **A** ****) The peptide DPT-C9 was administrated IP at 5 mg/kg once daily, 5 days a week for 4 weeks in the K-Ras ^LA1^ adenocarcinoma mouse model, showing a significant decrease in lung tumour burden compared to control formulating vehicle-treated mice (p = 0.01). **B**) Histological analysis of lung tumours of control treated only with the formulating vehicle and DPT-C9 -treated mice. **C**) DPT-C9 was administrated IP as for the K-Ras^LA1^ model in mice bearing xenografted mouse PyMT breast tumours, with a significant TGI of 46% after 11 days of treatment compared to control mice treated with the formulating vehicle. **D**) DPT-C9h was administered IP at 1, 5, or 25 mg/kg once daily for 5 weeks in mice bearing HBCx-12A tumours (triple negative model). Ten mice were included per group and the control group was treated with the formulating vehicle. **E**) DPT-sh1 and DPT-C9hM was administered IP at 1.5 mg/kg and 5 mg/Kg respectively, once daily for 5 weeks in mice bearing HBCx-12A tumours generated from the HBCx-12A cell line. Ten mice were included per group. **F**) DPT-C9h was administered IP at 5 mg/kg in mice bearing HBCx-12A cell line previously infected with a Ds-Red-Luc+ lentivirus. Bioluminescence imaging was shown in two mice (out ten), one receiving control vehicle (right mouse) and the other treated by DPT-C9h (left mouse). **G**) DPT-C9h was administrated IP at 5 mg/kg in mice bearing HBCx-3 (luminal model) once daily for five weeks. Ten mice were included per group. **H**) Relative variation of all treated tumours. In all *in vivo* experiments, mice of the control groups received 0.2 ml of the drug-formulating vehicle with the same schedule as the treated animals. Growth curves were obtained by plotting mean RTV against time. When RTV of all treated mice were considered from positive ration (resistant tumours) to negative ratio (sensitive tumours), we observed that 72% of all 198-treated mice have negative ratio, showing that peptide treatment has a high *in vivo* anti-tumour effect in BC xenografted models.

We further analyzed the potential anti-tumour effect of the peptide DPT-C9h using human breast cancer models. Using human breast cancer xenografts, we first treated mice bearing the triple negative breast cancer model HBCx-12A [27]. DPT-C9h was intraperitoneally administered at 1, 5, or 25 mg/kg, once daily for 5 weeks. At the end of the treatment, we observed that DPT-C9h induced significant tumour growth inhibition (TGI) of 50% (p<0.04), 37% (p<0.11), and 48% (p<0.04) according to previously defined doses and, compared to control mice treated with the formulating vehicle alone (Fig 6D). As negative control, DPT-sh1 or DPT-C9h mut were administered to mice bearing HBCx-12A at 1.5 mg/Kg and 5 mg/kg respectively, without any inhibition of tumour growth *in vivo* (Fig 6E). This result strongly suggests that the inhibition observed is due to competition by the binding motif since the shuttle alone or a mutated binding sequence did not have any effect. In order to validate antitumoral efficiency of DPT-C9h through optical imaging, we used the HBCx-12A cell line, derived from the HBCx-12A xenograft, infected by Ds-Red-Luc+ lentivirus to generate the xenograft model. DPT-C9h was administered at a dosage of 5 mg/kg daily for 4 weeks. Using optical imaging, we showed that DPT-C9h inhibited tumor growth of HBCx-12A cell line compared to control non-treated group that receive only the formulating vehicle (Fig 6F), as previously observed (Fig 6D). We conclude that the breast xenograft model obtained directly from the tumour or the breast xenograft generated from the cell line HBCx-12A respond equally to DPT-C9h treatment.

Similarly, DPT-C9h was tested in the HBCx-3 xenograft model. DPT-C9h induced an optimal and significant TGI in the luminal B breast cancer HBCx-3 model (85%; p<0.02) (Fig 6G). Interestingly, in this luminal breast cancer model, DPT-C9h induced 12 complete remissions in the 39 treated mice (31%) (p<0.01), in which 5 were prolonged after 2 months. Finally, to evaluate responses to DPT-C9h or DPT-C9 peptides according to individual mouse variability, and show peptides efficacy using waterfall plot representation, we decided to consider each mouse as one tumour-bearing entity. In each *in vivo* experiment, an individual response was defined for each treated mouse from the following formula: 1**−**(Vt/Vc), where Vt is the volume of the treated mouse and Vc the median volume of the corresponding control group at a time corresponding to the end of treatment. When considering positive ratio (resistant tumours) and negative ratio (sensitive tumours), we observed that 72% (41%+31%) of all 198 DPT-C9h/DPT-C9-treated mice had a negative ratio. From the 72%, 31% had a ratio lower than 50% and 41% a ratio higher than 50%, respectively (Fig 6H), showing that both peptides have a high anti-tumour effect in xenografted breast cancer models. Taken together, our results show that breast cancer models, triple negative, luminal, lung K-Ras mutated and PyMT respond to DPT-C9h or DPT-9 treatment showing considerable tumour growth inhibition.

## Discussion

In this report, we have demonstrated the interaction between caspase-9 and the serine/threonine phosphatase PP2A. We have generated a new cell penetrating peptide that specifically binds to PP2Ac (DPT-C9h or DPT-C9), targets caspase-9/PP2Ac interaction, leading to caspase-9 activation, mitochondrial membrane permeabilization, cytochrome *c* release and apoptosis in a variety of human and mouse cancer cell lines. In addition, the peptide specifically induces apoptosis in tumour cells, without effect on healthy primary cells. DPT-C9 and DPT-C9h also inhibit tumour growth in mouse or primary human breast cancer models. Finally, this peptide was not immunogenic and not toxic in *nude* mice implying that it multiple doses can be administrated without nullifying antibodies being generated.

Cell penetrating peptides have been evaluated for their ability to transport diverse cargos into cells, tissues, and organs. Few laboratories have targeted protein-protein interactions involved in anti-apoptotic signalling, including (i) the peptide shepherdin mimicking a small domain of the survivin protein that interacts with Hsp90 [34] (ii) peptides blocking PP1/GADD34 complex [35], [36], (iii) peptide inhibiting MUC1 interaction with EGFR [30], (iv) peptides with a sequence derived from elastine having the capacity to block invasion, migration and metastasis in ovarian tumours [37], (v) helix-stabilized cyclic peptides binding to estrogen receptor α and inhibiting ERα/coactivator interactions [38] and (vi) peptide (Tat) with a pro-apoptotic erbB2 sequence [39]. Similarly, several CPP are under clinical development, such as peptides targeting protein kinase c, Hsp20, and c-Jun-N-terminal kinase [40], [41], [42]. The promising results obtained in these studies indicate that CPP have an important role in the development of novel therapeutics. Moreover, an attractive feature of CPP is that they can specifically target a protein-protein interaction without affecting the rest of signalling pathways in which these proteins might be involved. In this report, we demonstrated that DPT-C9h targets the interaction between PP2A and caspase-9, without apparently affecting the rest of cellular PP2A, whose modulation might possibly induce toxicity.

It is known that PP2A is an important regulator of signalling pathways involved in oncogenesis, acting as a tumour suppressor complex. Recent work suggests that a specific PP2A complex regulates the activity of specific substrates, many of which are involved in cellular transformation [43], [44]. In breast cancers, PP2A has been reported to be involved in progression through various important signalling pathways; indeed, it has been reported that Her-2 receptor induced PP2A phosphorylation [45] that PP2A induced ERα dephosphorylation [46] and ERα mRNA instability [47], and that PP2A induced Akt dephosphorylation [48], [49], [50]. Moreover, it has been shown that interaction between PP2A and cofilin-1, a factor involved in actin polymerisation, increased cell motility and metastases. It is interesting to notice that while human and mouse PP2A share 98% identity, human and mouse caspase-9 share 72% of identity. There are four amino acids that differ between the binding motif, suggesting that these amino acids may be responsible for the species specificity and one could speculate that this sequence might be an interaction domain.

Given that human and mouse PP2A share an identity of 98%, it is intriguing to explain how human and mouse caspase-9 recognize differentially this protein. One hypothesis could be the presence of other proteins associated to the complex caspase-9/PP2A, which may regulate the access of the peptide to the protein-protein interface. Alternatively, different post-translational modifications between both species, such as phosphorylation or methylation, may result in the observed specificity.

In the same direction, and given that we have found similar amounts of complex caspase-9/PP2A in healthy and tumour cells (data not shown), it is exciting to understand how the peptide specifically recognizes tumour and no healthy cells. Our preliminary results show that there is a differential association of other partners to the complex caspase-9/PP2A between healthy and tumour cells which may explain this selective behaviour. All these data, combined to the specific targeting of caspase-9/PP2A interaction and the development of cell penetrating peptides as targeted therapies, support our innovative potential anti-tumour therapeutic approach. This penetrating peptide offers a promising approach specifically targeting tumour cells. In addition, selective activation of a signalling pathway leading to apoptosis of only tumour cells is the challenge in the development of new anti-cancer molecules.
